# Cardiac arrest triggers hippocampal neuronal death through autophagic and apoptotic pathways

This article has been retracted.

**DOI:** 10.1038/srep27642

**Published:** 2016-06-08

**Authors:** Derong Cui, Hanbing Shang, Xiaoli Zhang, Wei Jiang, Xiaofeng Jia

**Affiliations:** 1 Department of Anesthesiology, Shanghai Sixth People’s Hospital Affiliated with Shanghai Jiaotong University, Shanghai 200233, China; 2 Department of Anesthesiology and Critical Care Medicine, Johns Hopkins University School of Medicine, Baltimore, Maryland 21287, USA; 3 Department of Neurosurgery, Shanghai Ruijin Hospital Affiliated with Medical School of Shanghai Jiaotong University, Shanghai 200025, China; 4 Biomedical Engineering, Johns Hopkins University School of Medicine, Baltimore, Maryland 21205, USA; 5 Department of Neurosurgery, University of Maryland School of Medicine, Baltimore, MD 21201, USA; 6 Department of Orthopaedics, University of Maryland School of Medicine, Baltimore, MD 21201, USA

## Abstract

The mechanism of neuronal death induced by ischemic injury remains unknown. We investigated whether autophagy and p53 signaling played a role in the apoptosis of hippocampal neurons following global cerebral ischemia-reperfusion (I/R) injury, in a rat model of 8-min asphyxial cardiac arrest (CA) and resuscitation. Increased autophagosome numbers, expression of lysosomal cathepsin B, cathepsin D, Beclin-1, and microtubule-associated protein light chain 3 (LC3) suggested autophagy in hippocampal cells. The expression of tumor suppressor protein 53 (p53) and its target genes: *Bax*, p53-upregulated modulator of apoptosis (*PUMA*), and damage-regulated autophagy modulator (*DRAM*) were upregulated following CA. The p53-specific inhibitor pifithrin-α (PFT-α) significantly reduced the expression of pro-apoptotic proteins (Bax and PUMA) and autophagic proteins (LC3-II and DRAM) that generally increase following CA. PFT-α also reduced hippocampal neuronal damage following CA. Similarly, 3-methyladenine (3-MA), which inhibits autophagy and bafilomycin A1 (BFA), which inhibits lysosomes, significantly inhibited hippocampal neuronal damage after CA. These results indicate that CA affects both autophagy and apoptosis, partially mediated by p53. Autophagy plays a significant role in hippocampal neuronal death induced by cerebral I/R following asphyxial-CA.

Cardiac arrest (CA) affects nearly 300,000 and 450,000 people in the United States and Europe, respectively^1^,^2^. Advances in diagnosis and treatment have improved neurological outcomes after cardiopulmonary resuscitation (CPR). However, despite extensive experimental and clinical studies, numerous therapeutic trials have failed. Induced hypothermia improves survival and enhances the quality of neurologic recovery to the level of functional independence in 1 out of every 6 treated patients^3^, yet 5 out of every 6 treated patients continue to have poor outcome. Therefore, further research is needed to develop more effective measures to improve outcomes following CA.

Ischemia-reperfusion (I/R) injury following CA results in neuronal death by apoptosis and necrosis^4^, however, the molecular mechanisms are still unclear. Emerging evidence suggests excessive autophagy in several cerebral ischemic and neurodegenerative diseases^5^,^6^,^7^,^8^. However, its role in neuronal apoptosis remains to be elucidated. Autophagy may contribute to cell survival in some degenerative diseases via degradation of damaged and misfolded proteins. Conversely, excessive autophagy negatively impacts cell survival, thereby, causing cell death^9^,^10^,^11^. However, the mechanism underlying cell death remains unknown^12^,^13^,^14^. Increasing evidence, including the fact that several regulators are involved in both apoptosis and autophagy activation, suggests that autophagy and apoptosis are mutually influenced by each other in a complex interaction^15^,^16^,^17^,^18^.

Though the mechanisms that govern autophagy in cells are poorly defined, it is possible that mitochondria play a regulatory role in autophagy and apoptosis. Further, a few Bcl-2 genes such as *Bax* may mediate mitochondrial membrane permeability that subsequently triggers autophagy and apoptosis^19^. Bax triggers cell death. It plays a key role in tumor suppressor protein 53 (p53)-dependent apoptosis^20^. Reports suggest that p53 activates the transcription of Damage-Regulated Autophagy Modulator (DRAM), which in turn triggers autophagy as well as p53-mediated apoptosis^21^,^22^. Expression of *p53-upregulated modulator of apoptosis* (*PUMA*) triggers rapid apoptosis^23^,^24^. Compared with exogenous expression of p53, PUMA induces much quicker apoptosis^25^,^26^. Microtubule-associated protein 1A/1B light chain 3 (LC3) including LC3-II, which is translocated to autophagosomal membrane and is a known autophagy marker required for autophagosome formation^27^.

We reported previously that cerebral I/R increased NF-κB-dependent induction of p53 and autophagy. Preventing autophagy partially reduced pyramidal neuronal death, suggesting its role in ischemic injury^7^. However, whether p53 induction of autophagy in an ischemic brain following CA was adaptive, maladaptive, or mediated by cellular effectors common to apoptosis, is unknown. Autophagy is involved in both the promotion and inhibition of cell survival. However, the signaling pathways that regulate these cellular events remain poorly defined, underscoring the need for determination of other factors in autophagy and its impact on cell survival, specifically in the context of cerebral ischemia following CA.

In this study, we explored the role of autophagy involving hippocampal apoptosis triggered by global cerebral I/R injury following CA. Our findings may help elucidate the regulation of autophagy and cell death in CA. Furthermore, we identified new therapeutic targets for the inhibition of neuronal cell death and associated clinical therapeutic windows following CA for possible future clinical translation.

## Materials and Methods

### Animal Groups

This study was conducted following approval by the Animal Care and Use Committee of the Shanghai Jiaotong University (Shanghai, China), in accordance with the National Guidelines for Animal Experimentation and ARRIVE guidelines (Animal Research: Reporting *in vivo* Experiments). Male Sprague-Dawley (SD) rats weighing 300 to 350 g each were used (N = 6 per group, a total of 28 groups in 5 sub-experiments). The sample size was determined based on expected variances and differences between groups based on preliminary study. An additional set of 6 sham rats underwent similar surgical procedures excluding CA and CPR. Animals were individually housed with free access to water and rat diet and exposed to a 12 h light/ dark cycle, at 21 °C to 23 °C and 60% relative humidity.

To determine the expression and protein levels of LC3, p53, PUMA, Bax and DRAM, and evaluate the levels of lysosomal enzymes (cathepsin B and D) following ischemic hippocampal injury, rats underwent 8 min of CA after each group with specific drugs (as given below) administered before the CA experiment, were euthanized 1.5 to 24 h later, based on prior experiments. Rat hippocampi were dissected followed by RNA extraction and real-time PCR, or protein extraction for Western blotting analysis.

To observe the sequence of autophagy activation following CA, rats underwent CA and resuscitation and were euthanized at 1.5 h, 3 h, 6 h, 12 h, or 24 h after restoration of spontaneous circulation (ROSC). Transmission electron microscopy (TEM) was used to observe ultrastructural changes in rat hippocampal pyramidal neurons.

Biochemical evidence of autophagy activation was obtained in rats following CA at 1.5 h, 3 h, 6 h, 12 h, or 24 h after ROSC. Brains were removed, treated and stained. To determine whether p53 localizes to neurons, the hippocampal CA-1 region was stained for LC3 and NeuN or p53 and Beclin-1. To determine the differences in LC3 expression, the transcriptional levels of p53 and DRAM, Bax and PUMA following CA were examined. To further study the inhibitory effect of 3-MA on CA- associated changes in LC3-II, rats were pretreated with 3-MA (600 nmol) 10 min before the start of CA experiment and euthanized 3 h after ROSC, in comparison with CA-only animals at 3 h after ROSC and the sham animals. To study the inhibitory effect of E64 on CA-associated changes in LC3-II, sham animals were administered either E64 (900 μmol) or vehicle DMSO (5 μl) and euthanized 3 h later. Rats undergoing CA were administered with E64 10 min before the start of the CA experiment and euthanized 3 h after ROSC. The changes in cathepsin B, D and Beclin-1, p53 and DRAM, and Bax and PUMA following CA were examined.

To study the role of PFT-α on PUMA, Bax, DRAM and LC3-II following CA, rats were administered with PFT-α (30 nmol), PFT-α (60 nmol), DMSO (5 μl), or saline 10 min before initiating CA experiment and euthanized 6 h after ROSC.

To determine the role of PFT-α, 3-MA or BFA in the death of hippocampal neurons after CA, rats were administered with PFT-α (60 nmol), 3-MA (600 nmol), BFA (12 nmol), or DMSO 10 min before the start of CA experiment and were euthanized 7 days after ROSC. Thionine staining was used to estimate the number of intact pyramidal neurons in brain slides.

To determine whether 3-MA rescued hippocampal neurons from ischemic damage following CA, rats were exposed to DMSO or 3-MA (600 nmol) at 1.5, 3, or 6 h after ROSC and were euthanized 7 days after ROSC. Thionine staining was used to estimate the number of intact hippocampal pyramidal neurons.

### Intracerebroventricular cannulation

One week before CA, animals were cannulated in the left cerebral ventricle for i.c.v. administration of PFT-α, BFA or 3-MA as described previously^7^. The animals were anesthetized with an i.p, injection of 40 mg/kg 3% (v/v) pentobarbital sodium after appropriate cannulation as described previously (0.8 mm posterior, 1.4 mm lateral to bregma, and 4.0 mm ventral, Paxinos and Watson Rat Atlas) and verified using a Hamilton microsyringe to aspirate clear cerebrospinal fluid in microliter quantities. Four stainless steel screws were used to fix the guide cannula stabilized with acrylic dental cement. A dummy cannula was used during the recovery.

### Cardiac arrest and cardiopulmonary resuscitation

After fasting for 12 h with free access to water, animals were anesthetized with pentobarbital sodium, intubated and ventilated, following an i.v. dose of 2 mg/kg of vecuronium bromide, a neuromuscular blocker. The right femoral artery was cannulated for measurement of arterial MAP and arterial blood gases (ABG). These parameters, plus electrocardiographic recording, were measured before, during, and after CA. The right femoral vein was cannulated to administer drugs. A tympanic membrane temperature (Tty) probe was used to maintain Tty at 37.5 ± 0.2 °C using a lamp and heating pad. In our pilot experiments, Tty was within 0.4 °C of deep brain temperature under direct monitoring. The total surgical duration was approximately 20 min.

The CA and resuscitation protocols were conducted as reported previously^28^,^29^,^30^. Baseline measurements were recorded for 5 min after i.v. administration of 2 mg/kg of a second dose of vecuronium. The test drug was delivered into the left cerebral ventricle via the previously placed cannula. 5-min following the drug administration, a 5-min washout period was performed to avoid residue anesthetic effect. A third dose of vecuronium (1 mg/kg i.v.) was administered at the beginning of the washout period.

Asphyxia CA, defined by spontaneous MABP < 10 mmHg, was then induced by disconnecting the ventilator and clamping the tracheal tube. After 8 min of asphyxia, the tracheal tube was unclamped and resuscitation was initiated via mechanical ventilation, administering epinephrine and NaHC0_3_, and sternal compressions as previously reported^28^,^29^,^30^. At 60 min after ROSC, the rats were decannulated and transferred to a chamber containing 50% O_2_ for 30 min, and returned to their cages.

### Drug administration

All drugs (Sigma, St. Louis, MO, USA) were delivered through the cannula that was previously inserted into the lateral cerebral ventricle. The 3-MA (600 nmol), PFT-α (30, 60 nmol), E64 (900 μmol) and BFA (12 nmol) were mixed with 1% DMSO (Sigma, St. Louis, MO, USA) to a final volume of 5 μl, respectively.

### Electron microscopy and quantitative real-time PCR

Transmission electron microscopy (TEM) was used to observe the ultrastructural changes in hippocampal cells following CA, as previously reported^31^. Total RNA was extracted with the RNAiso Reagent kit and the cDNA was generated using the PrimescriptRT Reagent Kit (both from Takara, Dalian, LiaoNing China). The sequences of forward and reverse oligonucleotide primers specific to *LC3* (5′-CTT CGC CGA CCG CTG TAA-3′ and 5′-ATC CGT CTT CAT CCT TCT CCT G-3′), *p53* (5′-CCC AGG GAG TGC AAA GAG AG-3′ and 5′-TCT CGG AAC ATC TCG AAG CG-3′), *BAX* (5′-GCA TCC ACC AAG AAG CTG AG-3′ and 5′-CAA AGT AGA AGA GGG CAA CC-3′), *PUMA* (5′-GTG TGG AGG AGGAGG AGT GG-3′ and 5′-TCG GTG TCG ATG TTG CTC TT-3′), *DRAM* (5′-ATG GCC ATC TCC GCT GTT TC-3′ and 5′-TGG ATT CCA TTC CAG CTT GGT TA-3′), and rat glyceraldehyde-3-phosphate dehydrogenase (*GAPDH*) (5′-GAC AAT TTT GGC ATC GTG GA-3′and 5′-ATG CAG GGA TGA TGT TCT GG-3′) were designed using Primer5 software. Real-time quantitative PCR was examined with iCycler 5 (Bio-Rad, Hercules, California, USA). The Fast Start DNA Master PLUS SYBR Green I master mix (Roche Applied Science, Indianapolis, Indiana) was utilized to amplify a 20-fold dilution of each cDNA in a 20-μl volume, to obtain a final concentration of 200 nM for each primer. The PCR cycle conditions were 95 °C for 10 s, and 50 cycles of 95 °C for 20 s and 60 °C for 30 s. Melting curve analysis was used to evaluate the amplification specificity in a blinded fashion. Threshold cycle, Ct, was determined using the iCycler. The mRNA levels were normalized to GAPDH mRNA levels for each cDNA.

### Protein preparation and immunoblotting

Western blots were analyzed with homogenized and processed hippocampal tissues as we described previously^7^. Immunoblotting was conducted using the following antibodies: rabbit polyclonal anti-LC3 antibody (Abcam, Cambridge, MA, USA); goat polyclonal anti-cathepsin B antibody (Santa Cruz); goat polyclonal anti-cathepsin D antibody (Santa Cruz); mouse monoclonal anti-p53 antibody (Cell Signaling Technology, Woburn, MA, USA); rabbit polyclonal anti-PUMA antibody (Cell Signaling Technology); rabbit polyclonal anti-Beclin-1 antibody (Cell Signaling Technology); rabbit polyclonal anti-DRAM antibody (Assay Designs & Stressgen Bioreagents, Ann Arbor, MI, USA); and rabbit polyclonal anti-Bax antibody (Santa Cruz, CA, USA). Tissues were incubated in horse radish peroxidase-conjugated secondary antibody (anti-mouse, anti-rabbit or anti-goat IgG; 1:5000; Santa Cruz). After detecting the immunoreactivity with enhanced chemiluminescent autoradiography (ECL kit, Amersham, Arlington Heights, IL, USA) and normalizing to a GAPDH (Cell Signaling Technology) loading control, the levels of protein expression were quantified with Sigma Scan Pro 5 for comparison.

### Immunofluorescence analyses

Immunofluorescence analyses were examined as described previously^7^. Under deep anesthesia induced by an i.p. dose of 40 mg/kg of pentobarbital sodium, the rats were treated with PBS and 4% paraformaldehyde. The 30-μm-thick coronal brain sections were treated with antibodies against p53, Beclin-1 or LC3 (Cell Signaling Technology, Woburn, MA, USA) overnight, followed by FITC-coupled anti-rabbit IgG (Santa Cruz Biotechnology, CA, USA). The images were examined by an LSM 510 Meta confocal laser microscope. The immunoreactive signals were sequentially visualized with a fluorescence microscope (Eclipse TE 2000, Nikon, Japan) under high magnification (400×) with two distinct filters for dual-labeled sections. Quantification of p53, Beclin-1 or LC3 immunoreactivity was conducted in 10 microscopic fields (400×) each section in a blinded fashion. Three sections of ischemic hippocampus were analyzed ipsilaterally in each animal.

### Histochemical analyses

After transcardial perfusion with PBS followed by 4% paraformaldehyde perfusion under deep anesthesia, the brain tissues were processed, embedded in paraffin, and stained with thionine for routine histological studies. The total number of neurons in the hippocampus CA1 and CA3 region was examined blindly with Stereo Investigator software (MBF BioScience, Williston, VT, USA) and normalized to the control (sham group).

### Statistical analyses

Data are presented as mean ± SD. One-way analysis of variance (ANOVA), with Bonferroni post hoc test and Student’s t-tests, was performed to determine the statistical significance of data (GraphPad Software, San Diego, CA, USA). A p-value less than 0.05 was considered statistical significant.

## Results

Parameters and ABG levels. The physiological parameters (MAP, pH, and glucose) and levels of ABG including PaCO_2_ and PO_2_ were monitored before, during, and after (1 and 3 h post-ROSC) CA (Tables 1 and 2). All the observed parameters were similar across different animal groups with no significant difference.

### Autophagy activation in rat hippocampus following CA

The ultrastructure of brain tissues at various intervals after resuscitation was analyzed to identify hippocampal pyramidal neurons containing smooth cytoplasm, normal mitochondria (Fig. S1AA, black arrowheads) and nuclei. The pyramidal neurons showed autophagy or lysosomal activation and apoptosis following CA (Fig. S1AB–AF). Double-membrane structures or vacuoles (C-shaped) were seen in the autophagosomes (Fig. S1AB–AF, broad arrows), which were maximum at 3 h after ROSC (Fig. S1AC,AG). Fused autophagosome-lysosomes and phagocytosed organelles were present occasionally (Fig. S1AD, as indicated by asterisks). Swelling, blebbing, dilation, and broken cristae (Fig. S1AB, AC and AE, black arrowheads), along with a substantial decrease in intact mitochondria was observed (Fig. S1B). Darkly stained lysosomes showed phagocytosed lipids, as shown by narrow arrows in Fig. S1AC–AF. The organelles were lost and cytoplasmic vacuoles appeared 6 h after ROSC (Fig. S1AD). Cells also exhibited both apoptosis and necrosis 24 h after ROSC (Fig. S1AF). A significant increase in lysosomes was observed 6 h after ROSC (Fig. S1B).

The sequential changes in LC3 in the rat hippocampus following CA were monitored from 1.5 to 24 h after ROSC. The LC3 staining was indistinct in the CA1 subregion of the non-ischemic brains (sham group), while the staining was intense in the cytosol of hippocampal CA1 subregion showing a punctate appearance 3 h to 24 h after ROSC (Fig. S2). Abundant expression of LC3 mRNA was observed by quantitative real-time PCR, starting at 1.5 h with a peak at 3 h post-resuscitation (Fig. 1A). 3-MA pre-treatment significantly abrogated the LC3 mRNA expression at 3 h after ROSC (p < 0.05, Fig. 1D). LC3-I protein levels decreased 3 h after ROSC but increased subsequently. LC3-II protein levels were raised from 6 to 24 h after ROSC (Fig. 1B,C). At 3 h, LC3-I levels remained unchanged but LC3-II levels were greatly elevated, leading to a significant increase of LC3-II/LC3-I ratio (p < 0.05). This increase may be attributed to higher LC3 turnover as a result of robust autophagy activation.

Immunofluorescence staining showed that LC3 levels were relatively low in normal hippocampus but increased in the injured hippocampus between 3 h to 24 h after ROSC (Fig. S2) and the majority of hippocampal cells that stained intensely for LC3 protein (green staining) resembled neurons morphologically. Further, the increased expression of LC3-I and LC3-II was abrogated by the inhibitor of autophagy (3-MA) (Fig. 1E,F).

Autophagy activation was further assessed by monitoring the sequence of events in lysosomal enzymes cathepsin B, D and autophagy marker, Beclin-1, protein levels in rat hippocampus following CA at 3, 6, 12 and 24 h after ROSC. Increased activation of cathepsin B was observed following CA at 6 h and 24 h after ROSC (Fig. 2B,C). In contrast, the increase in lysosomal enzyme cathepsin D levels was observed between 3 and 12 h following CA and then significantly declined to a normal level at 24 h after ROSC (Fig. 2G,H). The protein levels of Beclin-1 also increased between 3 and 24 h after ROSC (Fig. 2A,F).

E64 inhibition of lysosomes was followed by an increased expression in hippocampal LC3-II in the sham treatment group, indicating the role of lysosomes in LC3-II degradation during autophagosomes maturation in a normal hippocampus (Fig. 2D,E). The increased expression of LC3-II following CA was also significantly enhanced by pretreatment with E64 (Fig. 2I,J), indicating that the turnover of autophagy was elevated after CA.

### Expression of p53 and its downstream factors in rat hippocampus increased after CA

CA is known to induce apoptosis. However, its effect on p53 expression has not been reported. We found a significant increase in p53 mRNA levels (Fig. 3A) following CA, starting at 1.5 h and peaking initially at 3 h after ROSC (Fig. 3B,C). Immunofluorescence assay using p53 antibodies (1c12) showed distinct p53 and Beclin-1 staining in the CA1 subregion of the non-ischemic brains (sham) and the staining was intense and the hippocampal CA1 subregion was marked by granular staining in cytosol at 3 to 24 h after ROSC. The p53 expression was localized to Beclin-1-positive pyramidal neurons in the hippocampal CA1 (Fig. S3).

The DRAM mRNA (Fig. 3D) and protein levels (Fig. 3E,F) increased from 1.5 to 24 h after ROSC, with a peak in mRNA expression at 12 h (Fig. 3D). We further assessed the p53 function by looking at its target genes, *Bax* and *PUMA*. *Bax* mRNA was expressed in the hippocampus 1.5 h after ROSC and peaked at 12 h after ROSC (Fig. 4A). The upregulation of Bax protein 6 to 24 h post-resuscitation with peaking at 6 h were observed (Fig. 4B,C). PUMA mRNA expression was observed 1.5 h after ROSC and peaked at 6 h after ROSC (Fig. 4D). Puma protein was upregulated at 3 to 12 h after ROSC (Fig. 4E,F).

### p53 inhibitor PFT-α inhibited autophagy activation after CA in rat hippocampus

The role of p53 inhibitor, PFT-α, on the expression of LC3 and DRAM in the rat hippocampus was investigated to determine the expression of p53 post-CA in neuronal autophagy activation. Pretreatment with PFT-α significantly inhibited the increase in *PUMA* and *Bax* mRNA and protein levels induced by CA, indicating blocked p53-mediated signaling (Fig. 5A–F). Similar inhibition of DRAM and LC3 (Fig. 6A–C), particularly LC3-II (Fig. 6D–F) mRNA and protein levels occurred following PFT-α pretreatment, suggesting the role of p53 in neuronal autophagy activation following CA.

### p53 and autophagy inhibitors attenuated CA-induced hippocampal neuronal death

In addition to p53 target genes in autophagy (*DRAM*) and apoptosis (*Bax*, *Puma*), we further investigated the role of PFT-α on the death of hippocampal cells following CA by thionine staining 7 days after ROSC. Further, we evaluated whether inhibition of autophagy by 3-MA or BFA contributed to PFT-α-mediated neuroprotection. We found that PFT-α treatment prior to CA substantially elevated the number of intact pyramidal neurons in the CA1 and CA3 areas 7 days after CA injury while CA alone resulted in substantial loss of the number of intact pyramidal neurons in the ischemic pyramidal layers of the CA1 and CA3 hippocampus at 7 days after ROSC (Fig. 7A,B). Both CA1 and CA3 hippocampal neurons were significantly increased in number after injury following 3-MA infusion prior to CA (Fig. 7A,B). Similarly, an increase in the number of intact hippocampal neurons of the CA1 and CA3 regions after CA was observed following pretreatment with autophagy inhibitor, BFA (Fig. 7A,B).

After an i.c.v. injection of 3-MA at 1.5, 3, or 6 h after ROSC, rats were euthanized 7 days later to evaluate the role of 3-MA in the rescue of the pyramidal neurons of the CA1 and CA3 hippocampal neurons from ischemic damage. The results showed that CA-induced hippocampal neuron damage was inhibited by i.c.v. injection of 3-MA only at 1.5 h after ROSC in the ischemic pyramidal layers of both CA1 and CA3 hippocampus (Fig. 7C,D).

Rats treated with 3-MA 1.5, 3, and 6 h after ROSC were euthanized 12 h after ROSC followed by immunofluorescence staining. LC3 staining was indistinct in the CA1 subregion of the non-ischemic brains (sham). At 12 h after ROSC, compared with the 3-MA -treated rats at 1.5 h after ROSC, the cytosol of the CA1 exhibited intense and punctuate staining in the vehicle-treated rats, and in 3-MA-treated rats at 3 h and 6 h after ROSC. The NeuN-positive pyramidal neurons in the hippocampal CA1 expressed LC3. The CA-induced hippocampal neuron autophagy was inhibited by i.c.v. injection of 3-MA 1.5 h after ROSC while no differences were observed between other groups and animals subjected to CA alone (Fig. S4).

## Discussion

The current study demonstrates that ischemic CA injury leads to cell death and increased autophagic activity, marked by accumulation of autophagosomes, autolysosomes, and other biomarkers. The increase in autophagosomes and LC3-II following CA is not likely due to decreased autophagic activity since an increase in active lysosomal cathepsins was also observed. Additionally, lysosomal inhibitor, E64, increased LC3-II expression, while class III PI3k inhibitor, 3-MA, decreased the levels of LC3-II.

Our findings further indicate autophagic mechanisms in hippocampal neuronal injury during cerebral ischemia following CA. An early decrease in the number of hippocampus CA1 pyramidal neurons has been reported after severe ischemic insults^6^,^7^. Our rescue studies demonstrated that 3-MA pretreatment within a critical time window of 1.5 h after ROSC inhibited apoptosis in hippocampal pyramidal neurons in both CA1 and CA3. No protection against hippocampal neuronal injury was observed at later time points. Thus, autophagy may mediates early signaling of cell death in hippocampal neurons. The interaction of autophagy with apoptosis and necrosis drives the cell to apoptotic or necrotic death, indicating that autophagy inhibition was ineffective.

CA induces apoptosis and necrosis concomitantly in hippocampus and cerebral neocortex^32^,^33^. However, the mechanisms underlying cell death and autophagy signaling are unclear. An increase in the number of double-membrane structures or vacuoles (C-shaped) were seen in the autophagosomes, starting 1.5 h after ROSC. Apoptotic features including disruption of cell membranes, chromatin pyknosis, and cell shrinkage and blebbing were observed in the later stages of recovery from CA. Previous animal study showed dramatically increased autophagosome formation and extensive hippocampal neuron death after H/I brain injury that was almost caspase-3-dependent, suggesting that autophagy plays an essential role in triggering neuronal death execution after H/I injury^34^. Our biochemical analysis was consistent with the morphological observations, with an increase in mRNA and protein expression of LC3, Bax, PUMA and cathepsins following CA, suggesting that cerebral I/R injury after CA triggers a variety cell death signaling molecules involved in apoptosis and autophagy.

Autophagic and apoptotic cell death are two forms of programed cell death that play crucial roles in the removal of unneeded and abnormal cells. While these two forms of programed cell death are morphologically distinct, recent studies demonstrate that autophagic and apoptotic cell death share some common regulatory mechanisms. Specifically, p53 participates in excitotoxic neuronal death, most likely through both apoptotic and autophagic mechanisms^35^. However, the role of p53 in the signaling pathway for autophagy and apoptosis during and after CA-induced brain damage is not clear. In the current study, we assessed the downstream mechanisms of p53 in mediating cerebral I/R injury following CA and showed that all tested proteins involved in autophagy including p53 and DRAM, Beclin 1, active cathepsin D and B, and LC3-II, were upregulated after CA. In addition, the test proteins involved in apoptosis showed increased expression of the pro-apoptotic p53 target genes PUMA and Bax after CA, with downregulation of the anti-apoptotic protein Bcl-2.

Our findings suggest that 3-MA, the BFA and PFT-α significantly and robustly inhibit both hippocampal cell death and the expression of autolysosome-related proteins induced by CA. PFT-α is a known small molecule inhibitor of p53 transcription activity while 3-MA is known as an autophagy marker^6^. Both autophaghy inhibitor 3-MA and lysosomes inhibitor BFA suppressed the autophagy and apoptosis activation after CA with improved neural survival, suggesting that the autophagy after CA might be upregulated and detrimental. In addition, the inhibition of p53 by PFT-α attenuated CA-induced autophagy and hippocampal neuronal apoptosis. These results are similar to those pre-treated with 3-MA. The PFT-α neuroprotection is likely responsible, at least partially, for the inhibition of autophagy. Thus, autophagy and apoptosis activation induced by CA may be dependent, at least partially, on a p53 mechanism. These results suggest that inhibition of p53 may inhibit both apoptosis and autophagic cell death, simultaneously. Therapeutic strategies to suppress autophagy-induced neuronal death might demonstrate the beneficial effects in the treatment of brain injury^34^. Therefore, p53 targeting might represent a neuroprotective intervention for various neuronal ischemic diseases. Further studies are needed to elucidate the detailed mechanism and to develop autophagic or p53-pathway targeted interventions to treat CA and to move this towards translational studies.

We sought to identify the role of p53 in hippocampal neuronal damage induced by cerebral I/R following CA. p53 is a known regulator of cell death and survival^7^,^31^,^35^. However, its role in hippocampal cell death during I/R following CA remains unclear. Recent studies demonstrate that a p53/Bcl-2 protein complex altered mitochondrial permeability, which resulted in cytochrome c release following transient global cerebral ischemia in rats^36^,^37^. However, the mechanism of mediation of neuronal apoptosis by the mitochondrial p53 pathway is unknown. Our results showed that CA led to the significantly increased expression of p53 mRNA and protein in rat hippocampus. We previously reported enhanced p53 expression and hippocampal neuronal damage 6 h to 12 h after carotid artery occlusion^7^. We now find that p53 expression and hippocampal neuronal damage increased rapidly 1.5 h after ROSC. These data suggest that p53 protein expression induced by cerebral I/R following CA in hippocampus promoted hippocampal neuronal damage.

p53 expression in apoptosis is well established^36^,^37^. Cell stress triggers p53 expression and multiple downstream target genes^32^,^38^. Our study shows that p53 induces the expression of pro-apoptotic protein Bax and the PUMA in the hippocampus. PUMA inhibits the interaction of p53 with Bcl-XL, which releases p53 that subsequently activate Bax^23^.

Recent studies suggest that p53 activates autophagy^7^,^31^,^35^. Our previous study reported that p53 triggered quickly a series of cell death signals and autophagy after focal cerebral ischemia. Inhibitors including SN50 and PFT-α prevent the expression of p53 and autophagy, thus reducing hippocampal neuronal injury^7^. The I/R-induced increases of protein levels of p53 and LC3-II, which reflects the excessive autophagic regulation with p53 upregulation and contributes to consequent apoptosis, were also significantly inhibited by treatment with 3-MA^7^. Crighton *et al.* showed that *DRAM*, a p53 target gene, was the inducer of cell death, and encodes a macro-autophagy inducing protein^21^,^39^. As an important gene for the enhancement of p53-dependent apoptosis, DRAM may enhance apoptosis induction via interaction with Bax and lysosome-dependent pathways^21^,^40^. Here we showed that the p53-specific inhibitor (PFT-α) and the autophagy inhibitor (3-MA) effectively inhibited the expression of *DRAM* and *LC3*-II, and hippocampal pyramidal neuronal death, suggesting that autophagy activation by p53 resulted in hippocampal neuronal death.

The role of CA in the injury of mitochondria is well recognized^41^,^42^. Mitochondria are the cellular energy sources. Therefore, cell membrane potential and structure are disrupted via mitochondrial dysfunction following CA^43^,^44^,^45^. Lysosomes are involved in cellular digestion and protease release. CA is linked to increased mitochondrial permeability and depolarization, mitochondrial release of pro-apoptotic granules, caspase-3 cleavage, and apoptosis^46^. Other apoptotic proteins including caspases and DNase released from Mitochondria suggested their major role in apoptosis^46^. However, it remains to be elucidated whether mitochondria plays a role in autophagy activation^11^,^47^,^48^.

Autophagic cell death was induced via mitochondrial electron transport chain complexes I and II^49^. Reports suggesting the role of p53 and autophagy in *in vivo* hippocampal cell death following CA are unavailable. Cerebral I/R injury that follows CA results in diminished energy metabolism, oxidative stress, and mitochondrial permeability^50^. We propose that autophagy is triggered by a decrease in mitochondria. The 3-NP induces striatal neuronal death following cytochrome c redistribution, temporary caspase-9, and calpain activation^51^. Our findings suggest that p53 regulated the expression of proteins mediating apoptosis and autophagy via interaction between autophagic and apoptotic pathways^7^,^52^.

The 3-MA inhibits translocation of cytochrome c in mitochondria to the cytosol during cell death induced by 3-NP^52^. Similar interactions in cerebral I/R-induced ischemic neuronal death were reported in our present and previous studies^7^. We already reported that autophagy induced degradation of Bcl-2^6^,^7^. Bcl-2 downregulation activates autophagy and apoptosis. Thus, Bcl-2 is crucial in the regulation of autophagic and apoptotic cascades that lead to neuronal death in dysfunctional mitochondria. The role of autophagy in Bcl-2 downregulation, cytochrome c release and caspase-3 activation, suggests that interaction between autophagy and apoptosis pathways might be common in cell death^53^.

Our findings suggest that 3-MA, the BFA and PFT-α significantly inhibit the hippocampal cell death induced by CA. PFT-α is a known inhibitor of p53 while 3-MA is known as an autophagy marker^6^. In addition, the inhibition of p53 attenuated autophagy and hippocampal neuronal apoptosis. These results are similar to those pre-treated with 3-MA. Previous studies have shown that p53 can also regulate necrotic cell death and autophagic activity mitochondria dysfunction including mitophagy^54^,^55^. Our findings may help elucidate the role of p53 in regulation of autophagy and cell death after CA. Though the sequence of these two critical processes may have a complicated interaction, our inhibition studies by p53 inhibitor showed downregulated autophagic regulation with improved neuronal survival, which may further support these hypotheses. The PFT-α neuroprotection is likely responsible, at least partially, for the inhibition of autophagy. These results suggest that inhibition of p53 may inhibit both apoptosis and autophagic cell death, simultaneously. Therefore, p53 targeting might represent a neuroprotective intervention for various neuronal ischemic diseases.

In conclusion, this study suggest that both autophagy and apoptosis mediate cell death following CA. Autophagy activation was partially mediated by p53, contributed to CA-induced hippocampal neuronal death, and preceded the apoptotic process. Further studies to identify the role of autophagy following CA are needed to elucidate the pathogenesis of cerebral ischemic diseases involving protein misfolding.

## Additional Information

**How to cite this article**: Cui, D. *et al.* Cardiac arrest triggers hippocampal neuronal death through autophagic and apoptotic pathways. *Sci. Rep.* **6**, 27642; doi: 10.1038/srep27642 (2016).

## Supplementary Material

Supplementary Information

## Figures and Tables

**Figure 1:** CA triggers LC3 mRNA and protein expression. Rats subjected to CA were euthanized 1.5 h to 24 h after ROSC and changes in LC3 expression were monitored. (**A**) LC3 mRNA upregulation; (**B,C**) Increased LC3 protein expression: Each bar denotes a ratio of LC3-II/LC3-I at different time points and represents mean ± SE; (**D**) 3-MA inhibited the CA-induced increase of LC3 mRNA levels at 3 h after ROSC; (**E–F**) Immunoblotting results showed that 3-MA abrogated the LC3-I and LC3-II increase at 3 h after ROSC. n = 6 per group. *p < 0.05 vs. Sham group, **p < 0.01 vs. Sham group; ^##^p < 0.01 vs. CA-treated group.

**Figure 2:** (**A–C, F–H**) Changes in Beclin-1, cathepsin (**B,D**) expression at different time points following CA. (**D–E**) Immunoblotting results showed pretreatment with E64 elevated LC3-II protein levels in sham-treated rat hippocampus. (**I–J**) Pretreatment with E64 enhanced LC3-II protein levels. n = 6 per group. **p < 0.01 vs. Sham group. ^#^p < 0.05 vs. Vehicle -treated group.

**Figure 3:** (**A–C**) CA upregulates p53 mRNA and protein levels. (**D–F**) CA upregulated DRAM mRNA and protein levels. Data represent percent of sham animals. n = 6 animals per group. *p < 0.05, **p < 0.01 vs. Sham group.

**Figure 4:** (**A,B**) CA triggered Bax mRNA and protein expression. (**C,D**) CA upregulated PUMA mRNA and protein levels. Protein bands normalized to GAPDH levels. Data represent percent of sham- animals. n = 6 animals per group. *p < 0.05, **p < 0.01 vs. Sham group.

**Figure 5:** (**A,B**) Inhibition of Bax mRNA and protein levels by PFT**-α.** (**C–E**) Inhibition of PUMA mRNA and protein expression levels by PFT-α. n = 6, *p < 0.05, **p < 0.01 vs. Sham group; ^##^p < 0.01 vs. Vehicle-treated group.

**Figure 6:** (**A,B**) PFT-α inhibited of CA-triggered upregulation in mRNA and protein levels of DRMA. **p < 0.01 vs. Sham group; ^##^p < 0.01 vs. Vehicle-treated group; (**C–E**) Inhibition of CA-induced increase in mRNA and protein levels of LC3 by PFT-α. n = 6. **p < 0.01 vs. Sham group; ^#^p < 0.05, ^##^p < 0.01 vs. Vehicle-treated group.

**Figure 7:** (**A,B**) Effects of 3-MA, PFT-α or BFA on hippocampal damage following CA. The treatment groups were as follows: (1) Sham treatment. (2) CA + DMSO treatment. (3) CA + 3-MA treatment. (4) CA + PFT-α treatment. (5) CA + BFA treatment. (**A,B**): Increased number of pyramidal neurons in the hippocampus after CA was observed in 3-MA, PFT-α, and BFA treated rats. (**C,D**) Effect of pre-treated 3-MA on hippocampal damage following CA. The treatment groups were as follows (1) Sham treatment. (2) CA + DMSO treatment. (3) CA + 3-MA treatment 1.5 h after ROSC. (4) CA + 3-MA treatment 3 h after ROSC. (5) CA + 3-MA treatment 6 h after ROSC. The number of hippocampal pyramidal neurons was substantially higher in the 3-MA-treated rats at 1.5 h after ROSC compared the vehicle-treated rats. Neuronal numbers were normalized to the sham group; n = 6 per group. **p < 0.01 vs. Sham group. ^##^p < 0.01 vs. Vehicle-treated group. Scale bar: 50 μm for higher magnification and 500μm for lower magnification in A and C, respectively. SO is for stratum oriens, SP is for stratum pyramidal, and SR is for stratum radiatum.

**Table 1:** Physiological parameters.

Groups	Time	MAP(mmHg)	pH	PaCO_2_(mmHg)	PO_2_(mmHg)	Glc(mg/dl)
Sham	Baseline	105 ± 5	7.36 ± 0.03	36.3 ± 3.6	142.3 ± 17.5	162 ± 26
	Asphyxia	103 ± 4	7.31 ± 0.02	38.8 ± 3.7	145.2 ± 17.6	171 ± 23
	ROSC 1h	106 ± 5	7.41 ± 0.02	38.5 ± 2.3	138.5 ± 16.3	169 ± 22
	ROSC 3h	104 ± 3	7.33 ± 0.03	39.5 ± 3.8	142.5 ± 18.2	173 ± 25
CA + DMSO	Baseline	105 ± 6	7.39 ± 0.02	39.2 ± 3.1	141.5 ± 14.6	172 ± 23
	Asphyxia	21 ± 3^a^	6.95 ± 0.03^a^	93.8 ± 6.6^a^	9.6 ± 5.2^a^	518 ± 27^a^
	ROSC 1h	96 ± 4	7.42 ± 0.08	35.8 ± 3.3	126.6 ± 15.5	353 ± 25
	ROSC 3h	93 ± 4	7.46 ± 0.07	36.5 ± 5.5	133.5 ± 14.1	286 ± 21
CA + 3-MA	Baseline	105 ± 8	7.45 ± 0.09	39.7 ± 2.5	140.2 ± 15.5	165 ± 26
	Asphyxia	22 ± 2^a^	6.85 ± 0.12^a^	98.2 ± 8.3^a^	6.5 ± 4.5^a^	491 ± 18^a^
(600 nmol)	ROSC 1h	113 ± 6	7.43 ± 0.10	38.3 ± 2.2	121.3 ± 16.1	339 ± 19^a^
	ROSC 3h	93 ± 6	7.48 ± 0.08	37.5 ± 4.2	138.5 ± 15.1	263 ± 21
CA + PFT-α	Baseline	96 ± 4	7.40 ± 0.06	39.5 ± 5.2	137.2 ± 18.2	158 ± 18
(60 nmol)	Asphyxia	20 ± 3^a^	6.89 ± 0.09^a^	95.3 ± 10.5^a^	8.3 ± 2.2^a^	465 ± 17^a^
	ROSC 1h	93 ± 4	7.38 ± 0.08	39.3 ± 6.2	125.1 ± 16.3	338 ± 21^a^
	ROSC 3h	100 ± 5	7.42 ± 0.05	37.5 ± 4.5	140.5 ± 18.1	223 ± 19
CA + BFA	Baseline	105 ± 6	7.39 ± 0.03	38.3 ± 3.6	141.3 ± 16.2	165 ± 18
(12 nmol)	Asphyxia	19 ± 4^a^	6.83 ± 0.12 ^a^	95.5 ± 6.9^a^	7.2 ± 16.6^a^	495 ± 15^a^
	ROSC 1h	92 ± 3	7.28 ± 0.13	36.6 ± 4.3	134.1 ± 13.9	369 ± 19^a^
	ROSC 3h	96 ± 5	7.46 ± 0.06	37.5 ± 5.5	139.5 ± 16.1	248 ± 20

All values are the mean ± SD. Arterial blood gas tensions include PaO_2_, PaCO_2_, pH and Glc. MAP, mean arterial pressure; PaO_2_, arterial oxygen pressure; PaCO_2_, arterial carbon dioxide pressure; Glc, glucose.

^a^Controlled parameter.

**Table 2:** Physiological parameters.

Groups	Time	MAP (mmHg)	pH	PaCO_2_(mmHg)	PO_2_(mmHg)	Glc (mg/dl)
Sham	Baseline	103 ± 6	7.33 ± 0.02	38.3 ± 3.7	143.3 ± 17.5	158 ± 19
	Asphyxia	105 ± 7	7.32 ± 0.03	37.7 ± 4.6	142.2 ± 18.3	161 ± 16
	ROSC 1h	107 ± 8	7.32 ± 0.03	39.5 ± 3.8	139.5 ± 17.6	159 ± 23
	ROSC 3h	108 ± 9	7.36 ± 0.04	38.9 ± 4.5	141.3 ± 16.8	162 ± 22
CA + DMSO	Baseline	105 ± 6	7.43 ± 0.03	39.3 ± 3.5	140.2 ± 15.5	159 ± 15
	Asphyxia	19 ± 3^a^	6.85 ± 0.08^a^	83.3 ± 13.3^a^	6.3 ± 4.1^a^	489 ± 18^a^
	ROSC 1h	100 ± 7	7.37 ± 0.06	38.3 ± 5.2	125.3 ± 15.5	338 ± 17^a^
	ROSC 3h	98 ± 9	7.46 ± 0.07	39.9 ± 6.1	138.8 ± 15.6	238 ± 16
CA + 3-MA 1.5 h	Baseline	106 ± 8	7.39 ± 0.02	40.5 ± 3.6	139.6 ± 15.3	165 ± 17
	Asphyxia	18 ± 5^a^	6.89 ± 0.07^a^	82.5 ± 11.6^a^	7.2 ± 3.5^a^	513 ± 18^a^
	ROSC 1h	112 ± 6	7.38 ± 0.06	41.6 ± 3.3	128.1 ± 15.9	343 ± 17^a^
	ROSC 3h	98 ± 7	7.45 ± 0.08	40.3 ± 5.2	132.3 ± 15.9	223 ± 15
CA + 3-MA 3h	Baseline	103 ± 9	7.40 ± 0.03	38.5 ± 3.8	140.3 ± 15.8	166 ± 17
	Asphyxia	20 ± 2^a^	6.89 ± 0.07^a^	80.1 ± 12.5^a^	6.6 ± 4.3^a^	568 ± 19^a^
	ROSC 1h	99 ± 7	7.36 ± 0.08	41.8 ± 7.2	129.5 ± 16.5	368 ± 25^a^
	ROSC 3h	95 ± 8	7.43 ± 0.06	38.7 ± 6.5	139.3 ± 15.5	253 ± 18
CA + 3-MA 6h	Baseline	107 ± 8	7.41 ± 0.03	39.3 ± 3.2	139.6 ± 16.5	168 ± 17
	Asphyxia	17 ± 6^a^	6.87 ± 0.08^a^	83.6 ± 13.5^a^	7.3 ± 2.8^a^	558 ± 19^a^
	ROSC 1h	103 ± 6	7.38 ± 0.07	39.8 ± 5.2	129.3 ± 16.3	362 ± 20^a^
	ROSC 3h	99 ± 7	7.45 ± 0.06	38.9 ± 5.6	133.3 ± 15.6	262 ± 18

All values are the mean ± SD. Arterial blood gas tensions include PaO_2_, PaCO_2_, pH and GlcI. MAP, mean arterial pressure; PaO_2_, arterial oxygen pressure; PaCO_2_, arterial carbon dioxide pressure; Glc, glucose.

^a^Controlled parameter.
